# Design and In Vitro Evaluation of Novel Cationic Lipids for siRNA Delivery in Breast Cancer Cell Lines

This article has been retracted.

**DOI:** 10.1155/2022/9231641

**Published:** 2022-06-06

**Authors:** Sandeep Vaidya, Manish Kumar Jeengar, Mohammad Ahmad Wadaan, Shahid Mahboob, Pankaj Kumar, Lisa M. Reece, Surender Reddy Bathula, Mycal Dutta

**Affiliations:** ^1^CSIR-Indian Institute of Chemical Technology (IICT), Centre for Academy of Scientific and Innovative Research (AcSIR), Hyderabad 500007, India; ^2^Department of Pharmacology, School of Pharmacy, Amrita Vishwa Vidyapeetham, AIMS Health Sciences Campus, AIMS Ponekkara, Kochi 682041, Kerala, India; ^3^Department of Zoology, College of Science, King Saud University, P.O. Box 2455, Riyadh 11451, Saudi Arabia; ^4^Integrated Regional Office, Ministry of Environment, Forest & Climate Change (MoEFCC), Government of India, Saifabad, Hyderabad 500004, Telangana, India; ^5^Reece Life Science Consulting Service, 819 N Amburn Rd, Galveston, TX, USA; ^6^Department of Pharmacy, BGC Trust University Bangladesh, Chittagong 4381, Bangladesh

## Abstract

Breast cancer is the most common cause of cancer mortality in Western nations, with a terrible prognosis. Many studies show that siRNA plays a role in the development of tumors by acting as a tumor suppressor and apoptosis inhibitor or both. siRNAs may be used as diagnostic and prognostic biomarkers in breast cancer. Antisurvivin siRNA was chosen as a therapeutic target in breast cancer treatment because it directly targets survivin, an inhibitor of apoptosis protein, that causes cell death. However, siRNA-based treatment has significant limitations, including a lack of tissue selectivity, a lack of effective delivery mechanisms, low cellular absorption, and the possibility of systemic toxicity. To address some of these issues, we provide a siRNA delivery method based on cationic lipids. In the recent past, cationic liposomes have displayed that they offer a remarkable perspective in proficient siRNA delivery. The presence of a positive charge plays a vital role in firm extracellular siRNA binding along with active intracellular siRNA separation and low biological adversities. Consequently, the methods for developing innovative cationic lipids through rendering and utilization of appropriate positive charges would certainly be helpful for benign and effective siRNA delivery. In the current study, an effort was made to synthesize a 3,4-dimethoxyaniline lipid (DMA) to improve the effectiveness and protection of successful siRNA delivery. DMA cationic lipid successfully delivered survivin siRNA that reduced the survivin mRNA expression, indicating the possibility of utilizing siRNA therapeutics for breast cancer. It is expected that this innovative quaternary amine-based liposome can open up new avenues in the process of developing an easy and extensively used platform for siRNA delivery. Cationic lipoplexes, a potential carrier system for siRNA-based therapies in the treatment of breast cancer, were proven by our data.

## 1. Introduction

With an estimated 39,510 deaths each year, breast cancer is responsible for 14% of all cancer deaths [1]. The ratio of cancer-related death and morbidity is growing every day due to various lifestyle and environmental factors [2]. This poses a great deal of concern for the developing nations with a large population like India, where the healthcare sector is inadequate and often inaccessible. After decades of cancer research, chemotherapy remains the first line of treatment which still lacks the efficiency of drug delivery to the specific target cells. As a consequence, normal organs and tissues are also exposed to the harsh environment of chemotherapeutic agents, causing dose-limiting adverse effects and toxicity, which is at the root of the therapy's failure [3]. It has been extensively studied that most cancers are the result of overexpression of cellular receptors or protein products [4].

Cationic liposomes are made up of cationic lipids with two hydrophobic aliphatic long chains and positively charged functions in their head groups. For usage as gene transfer vectors, cationic lipids are usually combined with neutral lipids such as dioleoylphosphatidylethanolamine (DOPE) or cholesterol (Chol). Cationic liposomes can create a charged combination with negatively charged siRNA molecules due to their opposite surface charge. The resultant charged lipid-siRNA complexes (often referred to as “lipoplexes”) are capable of efficiently delivering siRNA [5].

In recent years, cationic lipid-based siRNA therapy had an excellent contribution to the treatment of several diseases [6]. There are several reports on the use of cationic lipid-based gene delivery for treating diseases [7–9]. There are different viral and nonviral delivery vectors available. Due to the immunogenic effects of viral delivery vectors, they are not considered optimal compared to nonviral delivery vectors [10].

In the recent past, cationic lipid-based RNAi technology has been extensively explored and was found to bring the expression of certain oncogenes back to normal and put a halt to tumour growth [11]. There are instances in ovarian, prostate, and thyroid cancers where considerable progress has been made in developing siRNA therapeutics for these types of cancers, thereby paving a path for the treatment of other types of cancers too. The exceptional ability of RNAi's to fine-tune the expression of overexpressed cancer proteins allows this technology to be less oppressive on normal tissues and cells than standard chemotherapy [12]. The inability of antineoplastic drugs to effectively target tumor cells and their nonselective character are two key limitations of chemotherapy [13]. This demonstrates the urgent need to design a tumor-targeting delivery method for chemotherapeutic drugs that is both effective and safe. RNAi-based therapies are now being explored for a variety of disorders. Many RNAi-based medications are in clinical development, including patisiran, which targets the transthyretin (TTR) gene for treating hereditary transthyretin-mediated amyloidosis [14]. Keeping in view the great therapeutic potential that RNAi holds for clinical application, the present research is aimed at developing an effective delivery system that can successfully deliver siRNA into cells aimed at destroying the targeted oncogenic protein by degrading its mRNA.

## 2. Materials and Methods

### 2.1. Materials

All the reagents were purchased and were used without purification. Human survivin siRNA, agarose, MTT dye, penicillin/streptomycin antibiotic, and fluorescent siRNA were purchased from Sigma-Aldrich (St. Louis, MO, USA). The MCF-7, MDA-MB-231, and HEK-293 cell lines were gifted from the applied biology division, CSIR-IICT Hyderabad. Diethyl dicarbonate (DEP), solution of antibiotics (penicillin G, streptomycin, and amphotericin B solution), L-glutamine, and 3-(4,5-dimethylthiazol-2-ly)-2,5-diphenyl-tetrazolium bromide (MTT) were also purchased from Sigma. 18 : 1 TAP (dioleoyl-3-trimethylammonium propane (DOTAP)), polyethylene glycol (PEG), and cholesterol (Chol) were acquired from Avanti Polar Lipids, Inc. (Alabaster, AL, USA). HPLC-grade solvents like ethyl acetate, dicholoromethane (DCM), dimethyl sulfoxide (DMSO), and sodium sulphate (Na_2_SO_4_) were acquired from S.D. Fine Chemicals Ltd., respectively (Mumbai, India), and all the chemicals were used for workup and purification procedures.

### 2.2. Synthesis

The targeted compounds were synthesized using two steps. The comprehensive synthesis procedures and spectral data are shown in Supplementary Materials. All composites were analyzed by Fourier-transform infrared (FTIR) spectroscopy, hydrogen-1 nuclei nuclear magnetic resonance (1H NMR) spectroscopy, carbon 13 nuclear magnetic resonance (13C NMR) spectroscopy, and high-resolution mass (HRMS) spectroscopy. NMR spectra were verified on a Bruker 500 or 400 MHz system (Bruker, Billerica, MA, USA) in CDCl3 solvent. Chemical shifts for proton NMR were expressed in ppm level comparative to tetramethylsilane at 0 ppm. Chemical shifts for carbon NMR were expressed in ppm level relative to CDCl3 at 77.0 ppm. Data were described as chemical shift, multiplicity (s = singlet; d = doublet; dd = doublet of doublets; t = triplet; q = quartet), coupling constants (Hz), and integration. HRMS were documented from an Exactive™ Orbitrap high-resolution mass spectrometer with the Accela 600 UPLC system (ThermoFisher Scientific, Houston, TX, USA). The melting points of the samples were conducted on a Polmon MP-96 Automelt melting point apparatus (Polmon Instruments PVT LTD, Hyderabad, India). Column chromatography separation techniques were used for protein separation by silica gel (100–200 mesh). Infrared spectra were analyzed with a Bruker ALPHA FTIR spectrometer (Bruker, Billerica, MA, USA). Samples were thin films and expressed in cm^−1^ [15].

### 2.3. Scheme, Procedure, and Spectral Data of Synthesized Cationic Lipids

#### 2.3.1. Synthetic Scheme for the Synthesis of 3,4-DMA Lipid

Scheme for the synthesis of quaternized 3,4-DMA lipid is shown in Figure 1.

#### 2.3.2. General Synthetic Procedures for the Synthesis of 3,4-DMA Lipid

Synthesis of compound C is shown in Figures 1(a) and 1(c) The algorithm for the synthesis of compound C can be seen in Figure 1 [20]: (a) 3,4-DMA (1 mmol) and (b) potassium carbonate (4 mmol) were added together in a 250 ml round bottom flask containing ethyl acetate solvent (5 ml/gm) under an inert (N2 gas) environment and stirred for 10 min at room temperature. Next, 1-bromo alkyne chain (3 mmol) was added, and the mixture was allowed to reflux at 70°C for 48 hours. After 48 hrs, the reaction was checked by thin-layer chromatography (TLC) and mol wt. was confirmed by mass spec. (c) The mixture was then evaporated in a vacuum to eliminate solvents by diluting with water, evaporated by dichloromethane, and dehydrated with anhydrous sodium sulphate. The solvent was vaporized using a rotavapor evaporation system under pressure to obtain tertiary 3, 4-DMA lipid. Column chromatography was used for the purification of tertiary 3,4-DMA lipid with ethyl acetate/hexane as eluent [16]. Synthesis of compound D is shown in Figure 1(d). In the following reaction, tertiary 3,4-DMA lipid was liquefied in dichloromethane solvent and agitated for 10 min. Then, potassium carbonate and methyl iodide were added, mixed, and stirred for 12 hours at room temperature. After 48 hours, the reaction solution was analyzed by TLC, and mol wt. was confirmed by mass spec. The mixture was evaporated in a vacuum to eliminate solvents and unreacted methyl iodide, then diluted with water with the resultant lipid extracted with dichloromethane, and dehydrated in anhydrous sodium sulphate. The solvent was vaporized using a rotavap, under pressure to acquire the final product of quaternized 3,4-DMA lipid. Column chromatography was used for purification of the quarternized 3, 4-DMA lipid with ethyl acetate/hexane as the eluent. Characterization of this lipid was performed by HRMS, IR, 13C NMR, and 1H NMR (mentioned in Supplementary Information as analytical data 1.1) [16].

### 2.4. Formulation Development and Its Optimization

#### 2.4.1. Preparation of Liposomes

*(1) Ethanol Injection Method*. The ethanol injection method was adopted for making liposomes. Liposomes of 3, 4-DMA lipid were prepared using Chol, dioleoyl-3-trimethylammonium propane (DOTAP), and PEG by the ethanol injection method [17]. 3, 4-DMA lipid and Chol or lipid and PEG/DOTAP were dissolved in ethanol in different ratios, 1 : 1 and 1 : 0.5, and mixed properly. Next, various amounts of lipid (for making 1 mM, 0.5 mM, and 0.1 mM) were rapidly added into deionized water to make liposomes. For making liposome compound with DOTAP, cholesterol used a ratio of 1 : 1 (equal amount of compound and colipid), and PEG used 1 : 0.5 [18].

*(2) Preparation of Lipoplexes*. In this study, survivin siRNA was used for preparing lipoplexes. A fixed amount of siRNA (50 ng) and liposomes (25 *μ*M) were used for lipoplex formations. Charge ratios N/P of siRNA and liposome were 1 : 5, followed by the simultaneous measurement of size and zeta potentials (model: ZS90, Malvern, UK). Bath sonication (mode: POWERSONIC 405, New Delhi, India) was used to keep liposome particles from aggregating for more accurate size analysis [18].

*(3) Gel Retardation Assay*. The binding of siRNA with 3, 4-DMA liposomes was determined using 2% agarose gel. 3, 4-DMA liposome (25 *μ*M) was complexed with the siRNA (50 ng) at a cationic lipid : siRNA charge ratio of 5 : 1 in a total volume of 20 *μ*l and incubated on a rotatory shaker (model number: lab-200, Haryana, India) for 30 min. 6X loading dye (2 *μ*l) was mixed into each formulation sample, and the total solution was loaded into each well. The samples were electrophoresed at 100 V for approximately 30 min, and standardethidium bromide (EtBR) staining with UV fluorescent detection was employed, and the resultant image of the gel was captured using a GelDoc Go System (Bio-Rad Laboratories, Hercules, CA, USA) [19].

### 2.5. Cell Culture and Compound Preparations

Human breast cancer cell lines MDA-MB-231, MCF7, and the normal epithelial cell line HEK 293 (Cell lines were gifted from CSIR-IICT Hyderabad) were cultured in Dulbecco's modified eagle's medium (DMEM) (Himedia, Mumbai, India), supplemented with 10% fetal bovine serum (FBS, Gibco, Grand Island, NY, USA) with 1% pen-strep antibiotic solution in an incubator at 37°C with 95% humidity and 5% CO_2_. The standard solutions of mixtures were organized in absolute dimethylsulfoxide (DMSO) and diluted (stock concentration is 10 mM, and working concentration is 100 *μ*M to 1000 *μ*M) in culture media for further trials [20].

### 2.6. Cytotoxicity Studies

An MTT assay was executed to measure the cell viability of the treated cell lines. For the cytotoxicity experiments, 5000 cells per well were cultivated in 96 well plates and treated with different concentrations (ranging from 10 *μ*M to 1 nM) of 3,4-DMA liposomes for 48 hrs. After the end of the treatment period, the media was replaced with 90 *μ*l of fresh serum-free media and 10 *μ*l of MTT reagent (5 mg/ml) per well, and plates were incubated under standard conditions at 37°C for 4 h. Thereafter, the above media was replaced with 200 *μ*l of DMSO and incubated at 37°C for 10 min. The absorbance at 570 nm was measured on a Synergy H1 Hybrid Multi-Mode Reader (BioTek Synergy HT, Winooski, VT, USA) [21].

### 2.7. Intracellular Uptake Study

The intracellular uptake of siRNA by the cells was investigated utilizing a confocal microscope (magnification of 40x; model: FV1000, M/S Olympus, India) [16]. Almost 104–204 cells were seeded on poly-L-lysine-coated coverslips in six-well plates. Cells were treated with different optimized formulations: fluorescent siRNA, lipofectamine 2000 + fluorescent siRNA (10 *μ*l for 50 nM of siRNA, according to manufacturer's insructions), and liposome + fluorescent siRNA. After treatment, cells were fixed using 4% PFA, and DAPI (blue color) was employed for nuclear staining (20 min DAPI incubation). Cy5 (red color) was used to label the cells' siRNA. Coverslips were fixed on glass slides using mounting media and then sealed with paraffin wax [21].

### 2.8. In Vitro Gene Silencing Efficiency

Western blotting was used to define the proficiency of gene silencing within in vitro conditions [22]. The method works on the principle of separating proteins based on size, charge, and other differences in individual protein bands 105–205 cells were seeded in six-well cell culture plates. Cells treated with different optimized concentrations (lipoplexes were formed using an amount of siRNA (50 nM) and liposome (25 *μ*M) at a nitrogen/phosphate (N/P) charge ratio of 1 : 5) are as follows: (1) naked siRNA; (2) lipoplexes: (A) C12 : Chol (1 : 1) + siRNA, (B) C12 : DOTAP : Chol (1 : 1 : 1) + siRNA; (C) C12 : DOTAP (1 : 1) + siRNA, (D) lipofectamine 2000 + siRNA, (E) C12 : PEG (1 : 0.5) + siRNA and standard; (3) lipofectamine : siRNA (lipofectamine, 10 *μ*l, for 50 nM of siRNA). ImageJ (NIH, Bethesda, MD, USA) density measurement software was used for the analysis of the western blotting bands [23].

## 3. Results

### 3.1. Spectral Data of Synthesized Compounds

All the spectra of synthesized lipids are included in Supplementary Materials (Figures S1through S12).

### 3.2. Physical Evaluation of Cationic Liposomes

#### 3.2.1. Physical Characterization of Liposomes

The optimized formulation lipid product appeared to be clear, transparent, and homogeneous by macroscopic visual examination.

#### 3.2.2. Particle Size, Zeta Potential, and Polydispersity Index (PDI)

The size and charge of the self-assembled 3,4-DMA lipoplexes (siRNA:3,4-DMA complexes) were characterized by photon correlation spectroscopy/dynamic light scattering with a Malvern Zetasizer (model: ZS90, Malvern Panalytical, Malvern, UK). The results corresponding to all three lipoplex formulations are listed in Tables 1–3. All the graphs of size and charge are provided in Supplementary Materials (Figures S13to S20) [21].

### 3.3. In Vitro Studies

#### 3.3.1. Gel Retardation Assay

We prepared cationic liposomes of C10-3,4-DMA, C12-3,4-DMA, and C14-3,4-DMA lipids with DOTAP, Chol, and PEG (in the preparation of liposome ratio of compound and colipid is 1 : 1) as colipids by the ethanol injection method. These liposomes were used for making lipoplexes (liposome 25 *μ*M : siRNA 50 ng at a 5 : 1 charge ratio) by incubating siRNA and liposomes for 1 hr at 37°C [10]. As shown in Figure 2, C12-3,4-DMA : PEG liposome (25 *μ*M) : siRNA (50 ng) at a 5 : 1 charge ratio made the best complex (refer to Figure 2(b), yellow arrow). The C10 liposome cannot form any complex at 25 *μ*M with siRNA (50 ng), while C12 and C14 form complexes at 25 *μ*M. C12 with PEG also produced good complexation with siRNA.

#### 3.3.2. MTT Cell Cytotoxicity Assay

Gel retardation studies revealed that C12-DMA lipoplexes produced optimal complex formations (refer to Figure 2); hence, C12-DMA with various colipids was selected for further cytotoxicity studies on MCF7, MDA-MB-231, and HEK 293 (controls for the assay) cell lines. It was noted that the viabilities of the cells exposed to the various C12 lipoplexes were more biocompatible in comparison with the siRNA or liposome administered individually. The lipoplex formulations were made using Chol, DOTAP, PEG, and siRNA (50 nM) as discussed previously. Treatment was performed using different lipid concentrations from 1 nM to 1 *μ*M with the results showing that C12-DMA : PEG (1 : 0.5) lipoplex at IC50 of 0.2 *μ*M reflected good anticancer activity compared to lipofectamine or liposome alone (refer to data in Table 4). The comparative cytotoxicity findings are given in Table 4 (only 0.1 *μ*M concentration activity is shown in Table 4).

#### 3.3.3. Intracellular Uptake Result

The intracellular uptake of siRNA was evaluated by confocal microscope in the MDA-MB-231cells, and the results are illustrated in Figure 3. C12-DMA liposome (25 *μ*M) and fluorescent siRNA (50 nM) comprised the lipoplex. siRNA was Cy-5 labelled, and DAPI was used for nucleus counterstaining. The result shows that siRNA alone was not taken up into the cell, while C12-DMA : PEG (1 : 0.5) liposome at 25 *μ*M concentration successfully delivered siRNA into the MDA-MB-231 cell compared to lipofectamine and other lipoplexes.

#### 3.3.4. In Vitro Gene Silencing Efficiency

Western blotting shows the gene silencing efficiency of the optimized formulations (see Figure 4). Different lipoplexes were synthesized using C12-DMA lipid with DOT, Chol, and PEG colipids (25 *μ*M) and siRNA (50 nM), to evaluate the gene expression level in MDA-MB-231 cells. The results showed that C12-DMA : PEG (1 : 0.5) lipoplex completely decreased the survivin levels.

## 4. Discussion

At present, targeting mRNA and reducing the antiapoptotic protein expression in breast cancer using RNA interference is a powerful approach [24]. Delivery of siRNAs into cells is very difficult since these are highly hydrophilic and polyvalent anionic midsized molecules. The major rate-limiting factor of siRNA's therapeutic activity is poor accumulation in the target tissue due to its easy degradation in blood by nucleases [25]. It is essential to find an efficient drug delivery system for siRNA-based drug development. It is evident from several studies that cationic liposomes are considered suitable carriers for drug and nucleic acid delivery [26, 27]. Lower toxicity and immunogenicity, effective structural flexibility, better biocompatibility/biodegradability, and ease of large-scale preparation are advantages of a liposome-based drug delivery system [10].

Liposomes are generally considered to efficiently protect nucleic acids and allow uptake of these molecules by various cells [28, 29]. Based on this fact, 3,4-DMA cationic lipid was successfully synthesized and confirmed by IR, NMR, and HRMS. We have synthesized cationic lipid-based nonviral vectors of C10, C12, and C14 carbon chains containing 3,4-DMA cationic lipids for siRNA delivery. The siRNA binding characteristics of all the liposomes were evaluated by a simple gel retardation assay, and results indicate that the C10-DMA lipid cannot complex with siRNA very well; however, C12-DMA and C14-DMA successfully bound to si RNA. C12-DMA : PEG liposome (25 *μ*M) + siRNA (50 ng) at a 5 : 1 charge ratio developed the best complex for the uptake studies into cells.

For the cytotoxicity studies, C12-DMA liposomes were synthesized using Chol, DOTAP, and PEG complexed with siRNA. Results show that C12-DMA : PEG (1 : 0.5) lipoplexes delivered siRNA into the cell, so cell death will be more compared to lipofectamine and liposome alone.

Due to the cytotoxicity results, the C12-DMA liposome was selected for intracellular uptake studies (compound showing good efficacy in MDAMB-231 compared to MCF-7, so I choose MDAMB-231 for further study). Liposomes were synthesized using Chol, DOTAP, and PEG (25 *μ*M each) + siRNA (50 nM). The C12-DMA : PEG (1 : 0.5) liposome at 25 *μ*M concentration optimally delivered siRNA into the cells compared to lipofectamine and siRNA alone. To extend the delivery potential of these liposomes when coupled to siRNA, we transfected cancer cells with the siRNA complexes. Western blots confirmed that C12 : PEG (1 : 0.5) liposomes efficiently transfected siRNA into the breast cancer cell lines MDA-MB-23. As evident by MTT results, naked siRNA was unable to show significant cytotoxicity towards both of these cell lines, indicating the need for a carrier for successful uptake of siRNA, confirming most of the data seen in the literature [30]. We compared the efficiency of siRNA transfection using our liposomes C12 : PEG (1 : 0.5) and the commercially available reagent, Lipofectamine 2000, a well-known reagent used for transfection. Our results revealed that siRNA delivery by C12 : PEG (1 : 0.5) liposomes was more efficient than that obtained by Lipofectamine 2000 or any of the other synthesized liposomes. C12-DMA liposomes with PEG showed optimal intracellular delivery compared to lipofectamine and other lipoplexes. The absence of specific cell targeting by liposomes, however, is the often reported limitation of their use [31, 32]. To ensure the safety and selectivity of these lipoplexes towards cancer cells, we further performed MTT assays on the normal human embryonic kidney cell line (HEK 293) and the breast cancer cell lines, MDA-MB-231 and MCF-7, and found that treatment with C12 : PEG (1 : 0.5) with siRNA was highly selective toward the cancer cell lines tested when compared to the normal HEK 293 cells.

We have also evaluated the endogenous gene silencing efficiency of survivin siRNA delivered by C12-DMA liposomes in MDA-MB-231 cells by western blot. Survivin is a member of the inhibitor-of-apoptosis (IAP) family of proteins and is overexpressed on breast, prostate, and colon cancer cells. Survivin plays a key role in regulating cell division and apoptosis inhibition by blocking caspase activation [33]. Both survivin siRNA and C12-DMA liposomes with cholesterol and DOTAP alone did not completely inhibit protein expression levels of survivin because of a lack of spontaneous cellular entry. The C12-DMA lipoplex with PEG significantly decreased the survivin levels in MDA-MB-231 cells (compound showing good efficacy in MDAMB-231 compared to MCF-7, so I choose MDAMB-231 for further study) rendering the cells more prone to programmed cell death. It is important to note that the main finding of this work resides in substantiating the development of our C12-DMA liposome as a new class of drug delivery vector by successfully delivering survivin into breast cancer cells.

Lipid-based drug delivery systems provide a concrete platform for effective and specific drug delivery in many diseases where other delivery systems have failed [19, 34]. The advantages offered by the lipid delivery systems in carrying the active constituent to the site of action need to continuously be explored and established [35]. Several cationic lipids are available on the market for nucleic acid delivery, so we synthesized a cationic lipid that contains a positive charge, thereby successfully delivering siRNA into two breast cancer cell lines. We found that C12-DMA : PEG lipoplex produced better transfection activity than the marketed Lipofectamine 2000 lipid. These preliminary results of the biological screening of the tested liposome-siRNA treatment could offer hopeful support in this field and may lead to the discovery of a novel potent anticancer agent.

## 5. Conclusion

In the present research, a successful attempt was made in developing a highly selective and efficient cationic lipid-based siRNA delivery system. In the treatment of breast cancer, a cationic lipid (3,4-dimethoxy aniline was modified into a cationic lipid) based delivery method was designed to condense siRNA into antisurvivin-containing lipoplexes. Lipoplexes containing antisurvivin siRNA (C12 : PEG (1 : 0.5) and siRNA) delivered siRNA to MDAMB 231 cells with considerably better efficiency than other lipoplexes or lipofectamine alone did in vitro. This molecule-based strategy of siRNA delivery suggests that this lipoplex formulation has the potential to be used in the development of siRNA-based therapies. and it is more selective than the existing anticancer therapies by enhancing target-specific drug delivery for the treatment of breast cancer.

### 5.1. Statistical Analysis

All results were expressed as mean ± SEM (standard error of the mean). The in vitro data were analyzed for statistical significance using one-way ANOVA followed by Bonferroni multiple comparison procedure (Prism software, version 5.0; GraphPad Software, San Diego, CA, USA). Results were considered statistically significant when *p* < 0.05.

## Figures and Tables

**Figure 1:** Scheme for the synthesis of quaternized 3,4-DMA lipid.

**Figure 2:** Gel retardation study was carried out using standard gel electrophoresis. (a) Well 1: naked siRNA (50 ng); well 2: C10 : Chol (1 : 1) + siRNA; well 3: C10 : DOTAP (1 : 1) + siRNA; well 4: C10 : DOTAP:Chol (1 : 1:1) + siRNA; well 5: C10 : PEG (1 : 0.5) + siRNA. (b) Well 1: naked siRNA; well 2: C12 : Chol (1 : 1) + siRNA; well 3: C12 : DOTAP:Chol (1 : 1:1) + siRNA; well 4: C12 : DOTAP + siRNA (1 : 1); well 5: C12 : PEG (1 : 0.5) + siRNA. (c). Well 1: naked siRNA; well 2: C14 : Chol (1 : 1) + siRNA; well 3: C14 : DOTAP:Chol (1 : 1:1) + siRNA; well 4: C14 : DOTAP (1 : 1) + siRNA; well 5: C14 : PEG (1 : 0.5) + siRNA.

**Figure 3:** Cy-5 siRNA transfection efficacy of the synthesized C12-DMA lipoplex on MDA-MB-231 cells. Lipo2000 was used as a control. Cy-5 expressions in cells are indicated by the red-orange fluorescence. DAPI nuclear staining is shown by blue fluorescence. The scale bar is 25 *μ*m.

**Figure 4:** Western blot results for C12-DMA lipoplexes. (A) Naked siRNA; (B) C12 : Chol (1 : 1) lipoplex; (C) C12 : DOTAP:Chol (1 : 1 : 1) lipoplex; (D) C12 : DOTAP (1 : 1) lipoplex; (E) lipofectamine 2000 + siRNA; (F) C12 : PEG (1 : 0.5) lipoplex. *β*-Actin was used as controls for the lipoplexes.

**Table 1:** Size, charge, and PDI of C10 3,4-DMA lipoplexes (C10 DMA liposome: siRNA).

Lipoplexes	Size (nm)	PDI (%)	Zeta potential (mV)
C10 : DOTAP (1 : 1)	402.2	27.2	56.1
C10 : DOTAP:Chol (1 : 1 : 1)	242.7	22.6	38.5
C10 : Chol (1 : 1)	335.0	25.9	20.1
C10 : PEG (1 : 0.5)	415.4	26.9	25.6

**Table 2:** Size, charge, and PDI of C12 M 3,4-DMA lipoplexes (C12 DMA liposome: siRNA).

Lipoplexes	Size (nm)	PDI (%)	Zeta potential (mV)
C12 : DOTAP (1 : 1)	228.7	27.9	25.3
C12 : DOTAP:Chol (1 : 1 : 1)	264.3	21.6	43.2
C12 : Chol (1 : 1)	301.5	25.1	24.6
C12 : PEG (1 : 0.5)	282.7	25.5	27.4

**Table 3:** Size, charge, and PDI of C14 M 3,4-DMA lipoplexes (C14 DMA liposome: siRNA).

Lipoplexes	Size (nm)	PDI (%)	Zeta potential (mV)
C14 : DOTAP (1 : 1)	239.9	21.8	26.1
C14 : DOTAP:Chol (1 : 1 : 1)	324.0	27.8	43.0
C14 : Chol (1 : 1)	319.3	6.5	38.5
C14 : PEG (1 : 0.5)	334.4	25.5	31.4

**Table 4:** Results of cell cytotoxicity studies on different cell lines.

Samples	Percent viability		
	MDA-MB231	MCF7	HEK 293
siRNA (50 nm)	98.23 ± 0.22	95.43 ± 0.17	94.65 ± 0.32
C12 : DOTAP (1 : 1)	78.27 ± 0.65	85.93 ± 0.33	90.31 ± 0.14
C12 : DOTAP:Chol (1 : 1 : 1)	87.31 ± 0.15	88.69 ± 0.14	95.45 ± 0.24
C12 : Chol (1 : 1)	81.26 ± 0.8	89.92 ± 0.15	91.14 ± 0.23
C12 : PEG (1 : 0.5)	72.25 ± 0.42	93.62 ± 0.24	96.15 ± 0.15
C12 : PEG (1 : 0.5) + siRNA (50 nm)	22.15 ± 0.55	30.59 ± 0.26	85.40 ± 0.30
C12 : Chol:DOT (1 : 1:1) + siRNA (50 nm)	41.69 ± 0.32	47.84 ± 0.32	78.62 ± 0.25
C12 : DOT:(1 : 1) + siRNA (50 nm)	48.25 ± 0.31	62.79 ± 0.11	80.24 ± 0.24
C12 : Chol (1 : 1) + siRNA (50 nm)	55.92 ± 0.65	70.50 ± 0.14	82.25 ± 0.14
siRNA + lipofectamine 2000	60.32 ± 0.44	65.48 ± 0.22	68.64 ± 0.13

## Data Availability

All relevant data are included within the article.

## Abbreviations

DEPC: Diethylpyrocarbonate
DMEM: Dulbecco's Modified Eagle Medium
DAPI: 4',6-Diamidino-2-phenylindole
ETBR: Ethidium bromide
FBS: Fetal bovine serum
MTT: 3-(4,5-Dimethylthiazol-2-ly)-2,5-diphenyl-tetrazolium bromide
Chol: Cholesterol
DOTAP: Dioleoyl-3-trimethylammonium propane
DOPE: Dioleoylphosphatidylethanolamine
PEG: Polyethylene glycol
DMA: 3,4-Dimethoxyaniline lipid
TLC: Thin-layer chromatography
DCM: Dichloromethane
DMSO: Dimethyl sulfoxide
mRNA: Messenger ribonucleic acid
siRNA: small interfering RNA.
